# Genealogical Clustering and Coordination Analysis of Knowledge-Driven Labor Competitiveness in the Context of Sharing Economy

**DOI:** 10.1155/2022/7357047

**Published:** 2022-05-05

**Authors:** Lou Yun

**Affiliations:** School of Economics and Management, Yiwu Industrial & Commercial College, Zhejiang, Yiwu 322000, China

## Abstract

In recent years, with the continuous development of information technology and the advent of the Internet + era, the sharing economy has not only changed people's life and consumption patterns but also reconstructed the value cocreation process between enterprises and customers. Unlike the traditional economic model in which the enterprise is the dominant player, in the sharing economy, the enterprise withdraws from the dominant position in the value creation process and becomes a platform to support and serve the value creation of users (customers in the traditional economic model), and users become the dominant player in value creation. Users are not only the core subject of value cocreation in the sharing economy model but also the key factor determining the profitability of enterprises and the image of the platform. Bilateral users create rich value for individual users, platform enterprises, and society through value creation behaviors such as trading of the right to use idle resources and online and offline communication and interaction. Therefore, it is necessary to study the value cocreation behaviors of bilateral users of shared service platforms. This paper studies the value cocreation of bilateral users of shared service platforms, hoping to help platform enterprises further understand user behavior and needs, better fulfill the role of support and service in the process of value cocreation, provide a good value cocreation environment for bilateral users, enhance the reputation and influence of platform enterprises through user value cocreation behaviors, expand market share, and form competitive advantages. This paper stands in the perspective of intellectual enterprises and studies the problem of knowledge sharing. From the perspective of individuals, it mainly analyzes the willingness and ability of individual knowledge sharing, focusing on the “prisoner's dilemma” in game theory to study the willingness of individuals to share. From the perspective of knowledge, we mainly analyze the interference brought by the implicit and exclusive nature of knowledge to knowledge sharing, focusing on the implicit nature of knowledge. In addition, this paper only studies the influence of value cocreation of consumer users on value cocreation of resource users and does not deeply explore whether the value cocreation of resource users influences the value cocreation of consumer users.

## 1. Introduction

By analyzing and organizing the existing domestic and foreign related researches on customer value cocreation under the sharing economy model, it can be found that there are mainly two limitations in the research on value cocreation in the context of sharing economy [1].On the one hand, among the existing researches, most scholars have analyzed the value cocreation process of travel platforms by selecting more typical platforms under the sharing economy model for case studies [2]. There are also scholars who analyze the mechanism of customer value creation under the sharing economy model [3]. The scope of existing research is almost focused on these few large platforms, while the application areas of the sharing economy are very wide, so the scope of research on value creation under the sharing economy model needs to be further expanded. On the other hand, the research perspectives are not sufficient [4]. First, scholars have mostly explored the influencing factors and mechanisms of value cocreation behavior from the perspectives of resource providers and resource demanders, respectively, but there are fewer empirical studies on the interaction effects of value cocreation between resource providers and resource demanders [5]. Second, the existing studies mainly focus on the motivation of value cocreation, the mechanism of value cocreation, and the role of users, but they do not analyze the impact of value cocreation. In view of this, this study takes bilateral users of shared service platform as the research object to explore the role of bilateral users' value cocreation on each dimension of customer value, and the relationship between resource users' value cocreation and consumer users' value cocreation, hoping to enrich and supplement the existing value cocreation theories [6].

Value cocreation has gradually become a popular research area in the past decade, and the research areas are mainly focused on value cocreation in the production field, value cocreation in the consumption field, and value cocreation in virtual brand communities, while the research on value cocreation in the sharing economy is still in its initial stage. Under the traditional economic model, enterprises dominate the value cocreation process, while under the sharing economy model, enterprises withdraw from the dominant position in the value creation process and become a platform to support and serve the value creation of users (customers in the traditional economic model), and users become the dominant players in value creation [7]. It also enriches and improves the empirical research results in the field of value cocreation in the sharing economy and is innovative to a certain extent. In contrast to the traditional economic model, users are the dominant value creators in the sharing economy, and in the sharing economy, the identity of users changes from being single demanders to resource providers (resource users) or resource demanders (consumer users) [8]. Due to the different identities of the leading value creators, scholars have mostly explored the influencing factors and mechanisms of value cocreation behaviors from the perspectives of resource providers and resource demanders, respectively, and have not only studied the influence between the value cocreation behaviors of bilateral users, but also insufficiently investigated the value outcomes resulting from the interaction of value cocreation between demand and supply users [9].In addition to investigating the impact of bilateral user value cocreation on customer value in the sharing economy platform, this paper further explores the impact of consumer user value cocreation on resource user value cocreation and the mediating role of resource user value cocreation between consumer user value cocreation and customer value [10]. It expands the research perspective of value cocreation under the sharing economy model with a certain degree of innovation [11].

At the same time, it takes a longitudinal view of the knowledge activities and business activities of each enterprise in the whole industrial value network to enhance the value-added effect of knowledge and improve the competitiveness of the whole industry. On the basis of combining the existing characteristics of manufacturing industry, this paper refines and improves the knowledge value chain model, conducts an in-depth study on its core competitiveness, analyzes the operation process of knowledge value chain based on manufacturing industry, studies the operation mechanism of the chain and the influence factors of core competitiveness, and constructs indicators to quantify the core competitiveness of enterprises by adopting the method of case study, so as to deepen the grasp of the essence of knowledge value chain of manufacturing industry. This study not only proposes new understanding and suggestions on the competitive advantage cultivation strategy of traditional manufacturing enterprises from the perspective of knowledge value-added but also has strong operability and theoretical significance for enriching and improving the theory of competitive advantage of enterprises based on knowledge value chain. This paper studies the value cocreation of bilateral users of shared service platforms, hoping to help platform enterprises further understand user behavior and needs, better fulfill the role of support and service in the process of value cocreation, provide a good value cocreation environment for bilateral users, enhance the reputation and influence of platform enterprises through user value cocreation behaviors, expand market share, and form competitive advantages.

## 2. Related Work

With the rapid development of sharing economy, different scholars have researched and discussed the business model in the context of sharing economy from different perspectives [12]. From the previous generalization of the concept of sharing economy, we can see that academics do not have a unified cognition of the concept of sharing economy, and the research on sharing economy platforms is even at the initial stage. The definition of sharing economy platforms cannot be obtained from the existing literature related to sharing economy, and the definition of sharing economy platforms stays at the stage of observation and description and is more inclined to summarize the functionality of platforms and statements with the help of cases, lacking a detailed definition of the essence of sharing economy platforms [13]. Researchers propose that a platform business model is a business model that connects two (or more) specific groups, provides them with interaction mechanisms, satisfies the needs of all groups, and subtly profits from them. From the platform's perspective, connecting different users on the platform increases the enterprise value of the platform and thus gains a competitive advantage [14]. From the perspective of platform users, the platform breaks the problem of information asymmetry in previous transactions for users, making it possible to precisely match supply and demand, greatly reducing transaction costs and realizing greater customer value [15].

The researchers propose that in the new model of collaborative consumption, the sharing economy platform has the functions of a traditional marketplace and breaks through geographical constraints [16]. The researchers argue that on the basis of breaking through the constraints of time and space, sharing economy platforms simultaneously play the roles of technology supporters and transaction coordinators. Researchers believe that the essence of sharing economy platforms is a new type of information intermediary supported by advanced information technology, emphasizing human participation and interaction and effectively connecting supply and demand resources [17]. In summary, the sharing economy platform is an intermediary business model in which the Internet supported by information technology is used as a link that breaks through geographical restrictions and connects users from different regions on a platform that not only provides them with interaction mechanisms, but also integrates resources and is transparent in terms of information so that users with different identities can be precisely matched and transaction costs can be reduced, while providing technical support [18].

This kind of sharing platform includes two kinds: one kind of resource users share resources through the platform as service-oriented resources [18]. The other kind of resource users provide corresponding services to consumer users while sharing resources through the platform, for example, travel sharing such as Drip, where car owners need to provide driving services to passengers while providing travel tools. In the case of travel sharing such as DDT, car owners need to provide driving services to passengers while providing travel tools, and landlords need to provide landlord-related services to tenants while providing living space [19]. Under the sharing economy model, resource suppliers with ownership of idle resources become resource users, who release information about idle resources through the platform, provide resource demanders with the right to use the resources, and obtain economic benefits [20]. The role of resource user is no longer played only by enterprises, but also by individuals, such as in the C2C business model [21]. In the transaction process, resource users not only gain economic benefits, but also build emotional ties and gain respect and a sense of accomplishment through the interaction with consumer users and optimize their social credit [22]. At the same time, due to the characteristics of the sharing economy, the user identities of resource users and consumer users can be switched depending on the demand for resources.

## 3. Workforce Clustering Analysis in the Sharing Economy

### 3.1. Characteristics of Customer Value in the Sharing Economy Model

In the traditional economic model, value creation runs through the interaction between enterprises and customers, and although the core is to create customer value, the value creation process is still dominated by enterprises, which determine the generation and supply of customer value. Under the sharing economy model, the enterprise withdraws from the leading position in the value creation process and becomes a platform to support and serve the value creation of users (customers in the traditional economic model), and users become the leading value creators. Users who own idle resources are transformed into resource users, and users who seek the right to use idle resources are transformed into consumer users. With the support of the platform, the process of sharing the right to use resources between resource users and consumer users through screening and matching is the process of value cocreation by bilateral users under the sharing economy model, and the collection of creating value by sharing the right to use idle resources is the realization of customer value under the sharing economy model. The formation process of customer value in the process of user value cocreation in the sharing economy model is modified by referring to the analysis of the value cocreation mechanism in the sharing economy model and combining it with its own research content, as shown in Figure 1.

Economic value mainly refers to the benefits obtained and costs saved by resource users and consumer users in the transaction process under the sharing economy model. For resource users, under the sharing economy model, they can not only earn economic income in the transaction by posting their personal idle resource information on the platform and trading the right to use goods or services, but also avoid the waste caused by idle resources to the greatest extent. For consumer users, under the sharing economy model, they no longer need to spend high fees to transfer ownership of goods or services, but trade the right to use goods or services at the lowest cost, reducing transaction costs and gaining economic value. The functional value is mainly reflected in the technical support received by resource users and consumer users during the whole transaction process of goods or services. The platform is the core element of the sharing economy, and the transactions of resource users and consumer users are completed with the technical support of the platform. The biggest change in the identity of customers in the sharing economy compared with the traditional economy is that customers change their identities from simple resource demanders to both resource users and consumer users, and they can change their identities at will. The platform not only supports the transformation of users' identities, but also provides technical support for resource users to publish information, consumer users to screen information, and bilateral users to match accurately. At the same time, it provides a safe and trustworthy environment for the whole transaction process.

Social value is the value embodied in the social relationship established between resource users and consumer users in the sharing economy model. First, bilateral users can interact to obtain the information they need and satisfy each other's social needs. Secondly, bilateral users revitalize a large amount of social idle resources through the process of sharing the right to use goods or services, thus saving social costs. Finally, bilateral users complete transactions through the payment system of the platform, optimizing the personal social credit of users.

In the sharing economy model, the user is the dominant customer value creator, and the identity of the user changes from a single demander to a resource provider (resource user) or a resource demander (consumer user). Due to the different identities of the dominant value creators, scholars have mostly explored the influencing factors and mechanisms of value cocreation behaviors from the perspectives of resource providers and resource demanders, but less empirical research has been conducted on the interaction results of value cocreation between demand-based users and supply-based users. It is found that the existing studies mainly focus on the motivation of value cocreation, the mechanism of value cocreation, and the role of users but do not analyze the value impact of value cocreation. In view of this, this study takes the bilateral users (resource users and consumer users) of the shared service platform as the research object to explore the role of bilateral users' value cocreation on customer value, and the relationship between consumer users' value cocreation and resource users' value cocreation and to study the mediating role of resource users' value cocreation in this process.

### 3.2. Value Cocreation Based on the Dominant Logic of Knowledge-Driven Labor Competitiveness

Value chain theory divides value-adding activities inside and outside the enterprise into two categories: basic activities and supporting activities. There are five types of basic activities: internal logistics, production and operation, external logistics, marketing and sales, and services. There are four types of supporting activities: infrastructure, human resources, technology development, and procurement management. This division of the value chain tells managers that not all activities in the production activities of any enterprise can be optimized to produce effects that distinguish it from other enterprises, but only improving the quality of certain specific activities has the ability to truly create value, and these activities can bring unique economic advantages to the enterprise and are the links in the enterprise value chain which need real attention. Similar to the value chain, the virtual value chain includes the process of collecting, organizing, screening, and distributing information, and enterprises carry out value-creating activities through different value chains. At present, value chain theory has developed to the stage of value network and global value chain, and value chain has become the key research object of enterprise strategic management. Scholars' discussions on value chain theory are roughly divided into the following categories. Based on the traditional value chain classification model, the value chain of an enterprise is further divided into internal value chain and external value chain. The internal value chain consists of basic activities such as production, sales, logistics, and service, while the external value chain consists of suppliers, the enterprise itself, distributors, and customers. The authors believe that only when the internal value chain and external value chain are closely linked and work together can value chain management improve the core competitiveness of an enterprise and achieve long-term growth of enterprise value, as shown in Figure 2.

In the process of enterprise value chain management, only certain specific activities in the enterprise value chain are the key links that enterprises need to pay attention to, these links form and create the strategic value of the enterprise, and value chain management is to emphasize that enterprises should seize these key links for strategic planning of the value chain and, at the same time, to achieve resource sharing and complementary strengths and weaknesses among various departments, so as to improve the differentiation of enterprise operation and help enterprises achieve competitive advantage.

The core of the knowledge value chain model lies in the value-added role of knowledge accompanied by business processes. The value chain link relies on a series of production creations in the enterprise's business process to obtain added value, and the knowledge chain link relies on the transmission, dissemination, dispersal, and sharing of knowledge elements to carry out the cycle of value-added knowledge. Since the production process of an enterprise is accompanied by the flow of knowledge elements, corresponding value-added knowledge can occur as the knowledge flow moves upstream and downstream in the value chain and eventually forms a multiple value-added structure. By studying and analyzing the key activities in the value-added process, it can help enterprises achieve the effect of sustainable innovation. The cyclic operation of the knowledge value chain in A1, A2, and A3 can help enterprises achieve knowledge innovation in the process of knowledge accumulation and integration in B1, B2, and B3, as shown in Figure 3. The integrated effect of the knowledge value chain model cannot be brought into play by the knowledge chain or value chain alone. When studying the knowledge value chain, we need to focus on its systemic nature so that the optimal effect of the knowledge value chain can be brought into play. By integrating the internal and external knowledge resources of the enterprise, it realizes the growth of the enterprise's technology, information, and knowledge resources and by talking about the transformation and output of these absorbed resources, the enterprise restructures and rebuilds the enterprise's knowledge business process while creating its own knowledge achievements.

In the shared service platform, confidentiality of user information and a safe and trustworthy transaction environment are the most basic needs of consumer users throughout the transaction process. In addition, resource users can provide more personalized goods or services by providing more specialization or based on the interests of consumer users, etc., which will increase the functional value of consumer users. Therefore, the cocreation behavior of resource users affects the functional value obtained by the cocreation behavior of consumer users. The consuming user creates a transaction relationship with the resource user through the screening of the desired resources. Before the transaction occurs, the consumer user further understands the resource information by communicating with the resource user, and under this interaction, a friendly and pleasant interpersonal relationship is created. And the information transmission and feedback behavior of resource users will further promote the interactive behavior of bilateral users.

In addition, in the transaction occurrence, the resource user creates a personalized consumption experience for the consumer user based on his or her interest, which will further promote the pleasure of the consumer user and thus increase the hedonic value. At the same time, bilateral users revitalize a large amount of social idle resources through the trading of goods or service usage rights, saving social costs, optimizing users' personal social credit, and realizing social value.

In the fitting process, the acquisition of the network parameters is essentially the problem of optimizing the nonlinear function, which is simply the problem of finding the best set of parameters *W*^*∗*^, *b*^*∗*^ that can satisfy the following:

(1) $$\begin{array}{c} W^{*},b^{*}=\underset{\min}{J}\left(W,q\right). \end{array}$$

The training loss function in this paper is as follows:

(2) $$\begin{array}{c} J_{\text{fix}}=L\left(\left\{p_{i}\right\},\left\{t\right\}\right). \end{array}$$

Linear interpolation for the *x*-direction:

(3) $$\begin{array}{c} f\left(R_{1}=\frac{x_{1}-x_{2}}{x_{1}+x_{2}}\right)=f\left(Q_{11}\right)+f\left(Q_{12}\right),\\ f\left(R_{2}=\frac{x_{1}+x_{2}}{x_{1}-x_{2}}\right)=f\left(Q_{22}\right)+f\left(Q_{12}\right). \end{array}$$

Then linearly interpolating in the *y* direction,

(4) $$\begin{array}{c} f\left(P\right)=f\left(x,y\right). \end{array}$$

In the shared service platform, consumer users, as resource demanders, choose the collaborative consumption model based on factors such as saving economic costs or pursuing personalized consumption experience. According to the demand for resources, they search and screen resources through the platform to find resource matches and complete transactions successfully.

### 3.3. Competitive Labor Force Table under Shared Services

The data collection of the pretest was in the form of a web-based questionnaire, and the link to this questionnaire was generated using the research platform and could be distributed by the web platform with the topic and by the friends around. A total of 150 questionnaires were collected for the pretest, excluding the extreme questionnaires with the same answers to all questions, of which 120 questionnaires were valid, and the recovery rate of valid questionnaires was 80%. The descriptive statistical analysis of the pretest sample is shown in Table 1.

Cronbach's *α* values were used to test the reliability level of the pretest sample scales. The measurement results are shown in Figure 4. The Cronbach's *α* values of each variable are higher than 0.7, indicating that the scales have high internal consistency. Second, the CITC values were used to verify whether the scale items needed to be deleted. The test results found that the CITI values of each question item were all higher than 0.6, indicating that the scale topics have a high degree of correlation.

The action process of knowledge value chain shows the characteristics of double-chain dynamics. In addition to the dynamic business process of the enterprise, knowledge is constantly being transferred and converted to each other inside and outside the enterprise. It is through the continuous cycle of knowledge activities that the knowledge reserve of the enterprise can be expanded, the knowledge value chain system can be continuously improved and enriched, and good conditions can be created for enterprise management. In addition, only by looking at the value flow and knowledge flow of the enterprise with a dynamic vision can we have a stronger grasp of the knowledge activities in the production operation of the enterprise. The systemic nature of the knowledge value chain refers to the characteristics of the correlative action of two chains. The two chains in the knowledge value chain model combine organically and operate systematically to form a circular closed system through the interaction of knowledge flow and value flow.

The value chain exists and acts on the business process of the enterprise, so that the enterprise can achieve incremental revenue by reducing cost. The essential difference with the value chain is that the knowledge value chain focuses on the intangible value creation of the enterprise on the basis of cost reduction, so as to achieve high quality and high level of value addition. Through the update of enterprise knowledge technology and information resources, enterprises can bring more excess value for themselves to enjoy, and this value reflects both financial value and the unification with knowledge value. Knowledge value can be expressed as explicit value, such as patent value and advanced equipment value, or intangible value, such as goodwill and word of mouth. The role of knowledge value chain is to systematically enhance the enterprise value and strengthen the overall competitiveness.

## 4. Coordinated Analysis of Labor Competitiveness

The value chain of an enterprise believes that any activity can first be done by inputting certain resources or elements, and after specific production and operation activities, the value of the enterprise is finally output. Based on this model, the knowledge value chain theory divides the whole enterprise activity process into three parts: input element, activity element, and output element. In the knowledge value chain model, the input element includes not only the material element input and human resource element input of logistics, but also the initial input of knowledge flow, and the knowledge element is the most important input element in the input element model. In the activity element, the enterprise performs a series of successive value creation, including material element creation and knowledge element creation, and finally forms a result with novelty and practicality. The output element carries out the output of results, which includes the process of intellectual and knowledge value transformation along with the output of finished products. Enterprise profit, employee value, customer value, etc. are integrated in the multiple value body of the output element and constitute the core competitiveness of the enterprise while forming the product.

The gender distribution of platform users is 56.1% male and 43.9% female, with a balanced ratio of male to female. The age distribution of people under 20 years old accounted for 18.7% of the total sample, while the population of users between 21 and 30 years old accounted for the most, reaching 43.50%, and those between 31 and 40 years old accounted for 22.24%, while users over 40 years old only accounted for 15.55%, concluding that the shared service platform is more in line with the selection preference of young people. In the distribution of education, undergraduate degree is heavier, reaching 50.39%, undergraduate degree accounts for 31.69% of the total sample, and the distribution of master's and doctoral degree accounts for 11.02% and 6.89%. In terms of income distribution, 21.65% of the respondents had a monthly income of less than 3000, 29.53% of the respondents had a monthly income of 3000–5000, and 31.69% of the respondents had a monthly income of 5000–7000. Among the respondents, 21.65% joined the platform for less than six months, 25.39% for six months to one year, 32.09 for one year to two years, and 20.87% for more than one year, so more than half of the users joined the platform for more than one year, which makes the data of this questionnaire have some guarantee for the research value. The average number of users visiting the platform less than 5 times per month accounts for 23.82%, 6–10 times accounts for 31.30%, 11–15 times accounts for 28.94% of the total sample, and the number of visits higher than 15 times accounts for 15.94%. The results of descriptive statistical analysis of the sample are shown in Figure 5. The resource user, as the platform individual to whom the consumer user is transacting, holds information about the resource user, which greatly affects the security of the transaction.

On the basis of input element, activity element, and output element, the knowledge value chain can be divided into two parts, value chain and knowledge chain, based on the theoretical subdivision of enterprise business activities and knowledge activities, and the process of activity element in the knowledge value chain. The value chain corresponds to the realistic production and operation processes of enterprises, including internal logistics, production and operation, external logistics, marketing and sales, and services; the knowledge chain matches the cycle of enterprise knowledge activities, from knowledge acquisition to knowledge absorption, knowledge sharing, knowledge application, and finally knowledge transformation. Knowledge acquisition refers to the perception and summary of enterprises and employees to knowledge carriers or external practical experience. The knowledge absorption stage is the initial internalization and recognition of the acquired contents, which is an important factor affecting the subject to give full play to the dynamics of knowledge creation. Knowledge sharing is to share and spread the acquired and absorbed knowledge, and the process of researching, testing, and using the knowledge can promote the proliferation of enterprise knowledge. The knowledge sharing stage usually has two indicators of sharing depth and breadth, which are generally reflected through software and hardware platforms as well as company measures. Knowledge application is the process by which enterprises internalize knowledge and thus form it into capabilities, experiences, technologies, and structures. Knowledge transformation is the process of transforming and applying knowledge theory to practice.

To ensure the accuracy of the findings, this study used SPSS25 software to test the reliability level of the sample scales using both Cronbach's alpha values and the coefficient of correlation between modified items and totals (CITC). The measurement results are shown in Figure 6. The Cronbach's *α* values of each variable and dimension are higher than 0.8, which indicates that the scales of each variable have high internal consistency. Second, the CITC values were used to verify whether the scale items needed to be deleted. The results of the test revealed that the CITI values of each question item were all higher than 0.7, indicating that each question of the scale has a high degree of correlation.

As an important characteristic that distinguishes an enterprise from other competitors, the core competitiveness of an enterprise is difficult to be imitated or copied by its rivals. The production mode, marketing mode, company culture, corporate philosophy, and talent quality of an enterprise form a unique value system, which support each other and synergize with each other to form the core competitiveness, thus determining the efficiency difference, revenue difference, company value, and development potential of different enterprises. As an enterprise's capability, core competency can be accumulated and precipitated to output a personalized and diversified corporate culture and corporate products that are acceptable to consumers, so that the enterprise can survive in the wave of competition and even become the benchmark of the industry by influencing other enterprises through subtle influence and inculcation. This study first used exploratory factor analysis to examine the structural construct validity of the scale. The results of the factor analysis passed the KMO test and Bartlett's spherical test, and the results are shown in Figure 7 with KMO = 0.57, *p* < 0.001, indicating that the latent variables have good structural validity.

Although different enterprises have different forms of core competencies, they are all the result of innovation, organization, and transformation of knowledge. Human capital is the carrier of knowledge with strong mobility, core technology is the result of scientific knowledge cohesion, enterprise culture is the tacit knowledge of self-improvement and self-innovation formed under the condition of long-term accumulation, and innovation ability is the recreation of knowledge and activation of enterprise wisdom. The management and organization ability, marketing ability, customer service ability, etc. are also another manifestation of enterprise knowledge and “wisdom.” In the background of knowledge economy, the core competitiveness can never be separated from knowledge, and it ultimately depends on the existing knowledge structure of the enterprise as well as the storage quantity and quality of knowledge and the ability of the enterprise to digest and absorb itself. Only continuous knowledge updating can consolidate core competitiveness, and only continuous knowledge planning is the strongest means of enterprise core competitiveness. In this study, AMOS23 software was used to conduct validated factor analysis on the variables. The results show that the factor loadings are all greater than 0.8, indicating that all of them are significant; the combined reliability (CR) values are all greater than 0.8, proving that there is good credibility among the observed variables of the same dimension and the intrinsic quality of the model is ideal; the average variance extractions (AVE) are all greater than 0.6, indicating that the observed variables can effectively reflect the potential qualities of their common factor dimensions and the convergent validity is ideal. The factor loading coefficients and AVE and CR values are shown in Figure 8.

In this study, common method bias was controlled procedurally by using measures such as ensuring anonymity and emphasizing the absence of right and wrong answers. The collected data were tested for common method bias using Harman's one-way test, and the results of the unrotated exploratory factor analysis extracted a total of four factors with eigenvalues greater than 1. The maximum factor variance explained was 33.68%, which did not exceed 40%, so the data in this study did not have serious common method bias and were within an acceptable range. This study used SPSS25 to perform correlation analysis of latent variables. The results showed that the value cocreation of resource users had a significant positive impact on economic value with a correlation coefficient of 0.880, on functional value with a correlation coefficient of 0.870, on hedonic value with a correlation coefficient of 0.887, and on social value with a correlation coefficient of 0.891; the value cocreation of consumer users had a significant positive impact on economic value with a correlation coefficient of 0.874, and the value cocreation of consumer users had a significant positive impact on economic value with a correlation coefficient of 0.874, correlation coefficient of 0.874, a significant positive effect on functional value with a correlation coefficient of 0.870, a significant positive effect on hedonic value with a correlation coefficient of 0.890, and a significant positive effect on social value with a correlation coefficient of 0.880 (where *p* < 0.01).

## 5. Conclusion

There is still room for in-depth exploration in the research content of this paper. First, this paper only explores the impact of value cocreation on customer value by bilateral users of shared service platforms and does not include enterprise platforms in the study, which makes the research results somewhat subjective. In addition, this paper only studies the influence of value cocreation of consumer users on value cocreation of resource users and does not deeply explore whether the value cocreation of resource users influences the value cocreation of consumer users. In future, researchers should further explore the interactive influence between them to enrich the theory of value cocreation. Analyzing from the main body of knowledge sharing, individual willingness to share and sharing ability are the main obstacles that cause knowledge sharing not to be implemented smoothly. For the willingness of individuals to share, I design the “willingness dilemma” of knowledge sharing by combining the principle of “prisoner's dilemma” in game theory and conclude that only through reasonable punishment and reward mechanism can the organization make the compensation gain when individuals share knowledge greater than the monopoly gain when they share knowledge exclusively, and then the individuals can share knowledge with each other. As for the sharing ability of individuals, the employees of intellectual enterprises have certain sharing ability, but intellectual enterprises pay more attention to improving this ability, and any individual needs to improve his or her ability to transfer and learn knowledge. This study not only proposes new understanding and suggestions on the competitive advantage cultivation strategy of traditional manufacturing enterprises from the perspective of knowledge value-added, but also has strong operability and theoretical significance for enriching and improving the theory of competitive advantage of enterprises based on knowledge value chain. In the future, the knowledge sharing among individuals can be realized only if the organization can make the compensation benefit when individuals share knowledge greater than the monopoly benefit when individuals share knowledge through reasonable punishment and reward mechanisms.

## Figures and Tables

**Figure 1:** The formation process of customer value in the cocreation process of user value in the sharing economy model.

**Figure 2:** Value cocreation in the dominant logic of knowledge-driven labor competitiveness.

**Figure 3:** Multiple value additions and enhancements.

**Figure 4:** Analysis of pretest results for each variable.

**Figure 5:** Descriptive statistical analysis of the sample.

**Figure 6:** Results of the reliability analysis of each variable.

**Figure 7:** KMO test and Bartlett's spherical test.

**Figure 8:** Factor loading coefficients and AVE and CR values.

**Table 1:** Descriptive statistical analysis of the pretest specimens.

Characteristic variables	Characteristic variables	Number of people	Percentage
Gender	Male	66	55
	Female	54	45
Age	<20	16	13.3
	20–40	84	70
	>40	20	16.7

## Data Availability

The data used to support the findings of this study are available from the corresponding author upon request.
